# Protection and Inheritance of Traditional Culture in Urbanization Construction Based on Genetic Algorithm under the Concept of Environmental Protection

This article has been retracted.

**DOI:** 10.1155/2022/5844732

**Published:** 2022-06-16

**Authors:** Lin Guo

**Affiliations:** Gannan Normal University, Ganzhou, Jiangxi, China

## Abstract

Chinese traditional culture is a typical “moral culture,” and traditional morality is the core and essence of culture. However, in recent years, the phenomenon of following the trend of rural construction has been particularly serious, and many villages have lost their original features. To solve the above problems, the genetic algorithm can be used to further explore the traditional culture of urbanization construction. A genetic algorithm is a natural evolutionary process that imitates natural selection and genetic operation in nature to obtain optimal solution, in which genetic operation mainly includes the processes of gene replication, crossover, and mutation. This paper studies the traditional culture of urbanization construction based on the genetic algorithm under the concept of environmental protection. Among the accuracy of urban construction land expansion, in 2018, the accuracy of ant colony algorithm, data mining algorithm, and particle swarm optimization algorithm is 58%, 51.8%, and 56.7%, respectively. The accuracy of this genetic algorithm is as high as 58.8%. It can be seen that the genetic algorithm in this paper has the highest accuracy in the expansion of urban construction land. Therefore, in the process of large-scale urbanization based on the genetic algorithm, we should pay attention to not being separated from traditional culture, not letting farmers lose their regional culture, local culture, and grassroots culture, and protecting the cultural-ecological environment on which these cultures depend.

## 1. Introduction

The original meaning of “culture” is “rule of culture” and “enlightenment,” that is, to influence and restrict people with ethics and etiquette and music rules and regulations. Chinese traditional culture is a typical “virtue culture,” and traditional morality is the core and essence of culture. However, in recent years, the phenomenon of following the trend of rural construction is particularly serious. Many villages have lost their original characteristics. The history and culture of countryside have also been damaged or even destroyed to varying degrees. This blind demolition and construction and disorderly development and construction pose a serious threat to the rural pattern and the historical style inherited for thousands of years [1]. At the same time, with the emergence of the word “nostalgia,” the local history and culture have been paid continuously more attention. China's urbanization construction is the core of the overall development of urban and rural areas and the carrier of the further expansion of industrialization. Urbanization construction should establish the concept of people-oriented and spatial balance, innovate the development mode, reflect and highlight the regional cultural characteristics of cities and towns, and promote the healthy development of urbanization construction with the construction of cultural characteristics. In the process of new urbanization, the specific methods of protecting and utilizing traditional culture are realistic and typical in Tibetan areas across the country. Therefore, through analysis and research on the protection and utilization of traditional culture in the process of new urbanization, it is of great and far-reaching significance to carry forward Chinese traditional culture and enhance the due historical status of Tibetan traditional culture [2, 3].

Under the concept of environmental protection, this paper analyzes the protection of traditional culture in urbanization construction and uses the optimization algorithm of the genetic algorithm to solve some problems of traditional culture in urbanization construction. A genetic algorithm is a natural evolutionary process that imitates natural selection and genetic operation in nature to obtain optimal solution. Among them, genetic operation mainly includes the process of gene replication, crossover, and mutation. Therefore, the operation process of the genetic algorithm is also the process of genetic variation of simulated genes and the calculation method of selecting excellent individuals through copying, crossover and mutation operations, and selection operations. As we all know, biological evolution is based on Darwin's biological evolution theory, and the next generation of biological groups is produced by the reproduction of the previous generation of biological groups. Therefore, the main content of the abstract genetic algorithm, which simulates the evolution process of organisms, is to simulate the evolution process of biological groups. In essence, the genetic algorithm is a direct search method that does not depend on specific problems. The genetic algorithm has been applied in pattern recognition, neural network, image processing, machine learning, industrial optimization control, adaptive control, biological science, social science, and so on. The main problem to be solved in the process of genetic algorithm operation is the chromosome coding method, which is the key problem of genetic algorithm implementation, the method of transforming optimal solution from solution space-to-gene space, and the gene expression of optimal solution [4]. The quality of solution transformation will affect the evolutionary efficiency and degree of optimization [5].

People in different regions and environments have gradually formed their own unique local culture and regional culture in the long-term production practice. The forms of expression include local drama, arts and crafts, folk stories, and handicrafts. Different regions have also shaped the cultural elements, such as the character and beliefs of the local people. Under the concept of environmental protection, the traditional culture of urbanization construction is studied based on the genetic algorithm. In the process of promoting the overall development of urban and rural areas, one of the policies and measures to implement industry-feeding agriculture and cities supporting rural areas is to promote industrialization and urbanization. Industrialization is an important part of economic development, and urbanization is the main carrier and driving force of economic development [6]. Through the genetic algorithm, the evaluation index system of urban renewal project transformation potential and the evaluation index system of urban renewal project transformation urgency under the concept of environmental protection are established, and then the location model of urban renewal priority transformation project is constructed from the perspectives of efficiency and fairness. With the help of the genetic algorithm, the location scheme meeting the actual needs is solved, which verifies the accuracy, scientificity, and operability of the model. It provides a practical basis for the transformation sequence of traditional cultural projects in urbanization construction. Urbanization itself is a process of cultural convergence. Therefore, in the process of large-scale urbanization based on the genetic algorithm under the concept of environmental protection, we should pay attention not to be separated from traditional culture, let farmers lose their regional culture, local culture, and grassroots culture, and protect the cultural ecological environment on which these cultures depend. The innovations in this are as follows:

1. This paper constructs the traditional cultural structure model of urbanization. The solution process of this model is similar to the evolution process of biological natural selection, and it is a process of iterative evolution from generation to generation. The fitness of individuals is calculated by fitness function, and proportion is divided on the wheel according to the fitness. Each individual is like a sector in the wheel, and a pointer is placed on the wheel to randomly select. The greater the fitness, the greater the probability of being selected, and the smaller the fitness, the smaller the probability of being selected.
2. The trend of the urban construction land expansion rate was tested and analyzed. From the perspective of the expansion rate, the growth rate from 2016 to 2021 showed the characteristics of first increasing and then decreasing. From 2016 to 2019, the expansion rate of urban construction land under the genetic algorithm reached 12% at the fastest, followed by 10% under the particle swarm algorithm, while the ant colony algorithm and data mining algorithm were only about 7% and 1%, respectively. It can be seen that the genetic algorithm in this paper is important in the expansion rate of urban construction land.

The overall structure of this paper consists of five parts.

The first chapter introduces the background and significance of traditional culture in urbanization. The second chapter mainly describes the research status of traditional culture in urbanization at home and abroad. The third chapter describes the principle and model of the genetic algorithm and the content of traditional culture protection and inheritance in urbanization. In chapter 4, simulation verification and analysis are carried out. The fifth chapter is a summary of the full text.

## 2. Related Work

### 2.1. Research Status at Home and Abroad

Guo et al. proposed that in the process of traditional urbanization, due to the lack of restraint mechanism for the protection and development conditions of rural cultural resources and the lack of attention to the scientific development of rural culture, rural culture is distorted and distorted, and the value of rural culture is greatly reduced [7]. Cheung et al. proposed that in the process of improving the appearance of villages, urbanization and ecological civilization, national unity, follow-up industry cultivation, spiritual civilization construction of farmers and herdsmen, and improvement of urban cultural connotation should be mutually promoted to reflect the characteristics [8]. Yang et al. proposed that the common development of urban and rural areas is an important premise and fundamental policy to narrow the economic and social gaps between urban and rural areas, and it is also the best choice to solve the contradictions and problems between urban and rural areas at present and in the future [9]. Liu et al. proposed that new urbanization has made a great change in the development of human society in Tibetan areas for thousands of years, so the protection and utilization of traditional culture is to inject new soul and add gorgeous color to it [10]. Li et al. pointed out that traditional culture is neglected in construction of urbanization, and there is a lack and dislocation of ideas for the construction of traditional culture [11]. Zhao et al. proposed that actively promoting the coordinated development of urban and rural areas is to establish a market system for the rational allocation of production factors between urban and rural areas, an effective system for the benign interaction of the urban and rural economy, and an operation mechanism for the common development of urban and rural social undertakings and infrastructure, and strive to eliminate the institutional obstacles to the coordinated development of urban and rural areas [12]. Zhang et al. proposed that market pursues the maximization of economic benefits. In the process of urbanization, it often pays too much attention to people's material prosperity, the development level of public cultural services is low, and even destructive development and utilization have caused irreparable losses to excellent traditional culture [13]. Li et al. proposed that rural urbanization should not blindly oppose the development strategy of big cities, or idealize the strategy of small towns, but should adopt diversified and low-cost development strategy to realize the all-round development of cities and towns, realize the low-cost of rural labor transfer to cities and towns, and the low cost of urban and urban construction, so as to facilitate the smooth transfer of a large number of rural labor [14]. Wang et al. proposed that the relevant elements with rural cultural resources as the core were not revitalized, resulting in the phenomenon of “foreign village” common, or the “one-time tourism consumption” of rural cultural products due to the rough utilization of relevant elements, which failed to extend the value chain of rural cultural resources [15]. Hakak et al. proposed that the overall protection and inheritance of traditional culture under the construction of new urbanization is based on the full excavation of regional material culture and intangible culture, so as to form a traditional cultural inheritance policy with clear protection direction and local characteristics through continuous efforts [16].

### 2.2. Research Status of This Paper

In this paper, the traditional culture of urbanization construction is studied based on the genetic algorithm under the concept of environmental protection. Traditional urbanization is not conducive to the protection, inheritance, and innovation of rural culture. In the process of new urbanization construction, the homesickness concept is used to guide the protection, inheritance, and innovation of rural culture, hoping to find a way to realize that the protection and development of rural culture complement each other, and inheritance and innovation keep pace with each other. Compared with rural areas, urban areas are more efficient, so we think that urbanization should be efficient in all aspects, including land conservation, but our urbanization is constantly devouring our land. The ultimate goal of the overall planning of urban and rural areas through the genetic algorithm is the integration of urban and rural areas, which is the advanced stage of modernization and urbanization, and the process of mutual absorption of advanced and healthy factors, rejection of backward and morbid conditions, mutual integration, and two-way evolution between urban and rural areas. On the basis of digging and protecting local history and culture in the genetic algorithm, rural development develops regional characteristic environmental protection industry, which drives rural development. However, completely copying or letting it develop is not conducive to the further advancement of urbanization in China. Therefore, it is necessary to take functional cultivation as foundation, cultural characteristics as the fulcrum, industrialization as the driving force, regional urban cluster construction, coordinated development of the large, medium, and small cities and small towns as the basic mode to make a good plan, and take the urbanization road of sustainable development in accordance with the principles of gradual progress, land conservation, intensive development, and rational layout. For the protection and inheritance of rural history and culture, a feasible planning method is put forward in the genetic algorithm under the concept of environmental protection, so as to protect the development space of environmental protection concept of Chinese history and culture, enhance its vitality, and have very important practical significance for carrying forward local culture and protecting the integrity of the Chinese nation's historical context.

## 3. Research Method

### 3.1. Principle and Model of the Genetic Algorithm

Genetic algorithm is an adaptive probabilistic search method, and the search process is based on global search. Its algorithm idea is similar to natural selection evolution. It is a simulation of biological genetic evolution in nature. It has penetrated into various fields of research and engineering with its strong problem-solving ability and wide adaptability, and achieved good results [17]. Genetic algorithm is a random, iterative, and evolutionary search method based on natural selection and population genetics. All natural species survive by adapting to the environment, which is the main law of the genetic algorithm. In the genetic algorithm, genetic operation mainly includes selection, crossover, mutation, and other operations. Through the change of some gene segments, biological genetic operation, and survival of the fittest in nature are realized [18]. In the operation process, some operation parameters will be involved, and the design of these parameters is generally randomly generated. Firstly, we determine the first-generation population, set the population number, and code it; we determine fitness function and calculate the fitness of population; optimal individuals are selected by the selection operator to form the next generation population, and individuals in the next generation population are cross-exchanged and mutated to form new individuals. When the number of iterations is completed, we search for the optimal individual output; otherwise, we continue the iteration. The flow of the genetic algorithm is shown in Figure 1.

#### 3.1.1. ① Choose

When the population size is set, if the value is small, the diversity of population will be lost, resulting in premature convergence and failure to reach optimal solution. However, if the value is too large, the operation time of the genetic algorithm program will be prolonged, which will affect the operational efficiency.

#### 3.1.2. ② Crossover

When the crossover probability is chosen, if the crossover probability is too large, it will affect the dominant gene inheritance of population itself, which is not conducive to the optimization of the whole population. However, if the crossover probability is too small, the generation speed of new individuals will slow down, and when the number of iterations reaches, optimal solution can still not be reached.

#### 3.1.3. ③ Variation

When mutation probability is selected, if mutation probability is too large, it will lead to too many gene mutations, which will make the difference between the new individual and the parent individual too large, thus losing the adaptive advantage of the genetic algorithm, resulting in the search process of optimal solution having no direction, and becoming the random search for optimal solution. However, if the mutation probability is too small, it will be difficult to generate new individuals, resulting in the generation of local optimal solutions [11].

When the impact on the result is positive, the data standardization formula is as follows:

(1) $$\begin{array}{c} A=\frac{A_{ij}-A_{j\min}}{A_{j\max}-A_{j\min}}. \end{array}$$

When the impact on the result is negative, the data standardization formula is as follows:

(2) $$\begin{array}{c} A=\frac{A_{j\max}-A_{ij}}{A_{j\max}-A_{j\min}}, \end{array}$$

where *A* is the standardized value of the index, *A*_*ij*_ is the actual value of the *j* index in the *i* year, *A*_*j*min_ is the minimum value of index *j*, and *A*_*j*min_ is the maximum value of *j* index.

According to the judgment matrix, the eigenvector *ω* corresponding to the maximum eigenvalue *λ*_max_ of the judgment matrix can be further obtained. The formula is as follows:

(3) $$\begin{array}{c} A\omega =\lambda_{\max}\omega . \end{array}$$

Then, the feature vector is normalized. The result of normalization is the ranking of the importance of corresponding index factors, that is, weight, *ω*=(*ω*_1_, *ω*_2_,…,*ω*_*n*_)^*T*^.

The transformation potential of the renewal project is evaluated, and the formula expression is

(4) $$\begin{array}{c} S=\sum_{i=1}^{n}f_{i}w_{i}. \end{array}$$

In the genetic algorithm, it is realized through the selection operator. The probability of individuals with high fitness to be inherited to the next generation population is relatively large, and the probability of individuals with low fitness to be inherited to the next generation population is relatively small. Finally, they continue to approach optimal solution. At the beginning of the development of rural tangible and intangible cultural resources by the genetic algorithm, it is necessary to clarify the constraints on the protection and development of rural cultural resources, that is, to find the constraints affecting the protection and development of rural cultural resources [19]. The development of cultural resources in this area through the genetic algorithm only provides preconditions for the development of rural cultural resources. If rural cultural resources need to be developed, it is also necessary to improve the function of elements, sublimate the function of elements, transform and optimize elements, and optimize elements. The traditional cultural structure model of urbanization construction is constructed, as shown in Figure 2.

The transformation potential of the urban land parcel can comprehensively and objectively measure the importance of urban renewal projects. The greater the transformation potential, the less difficult the transformation of the urban land parcel and the greater the benefits. The potential of urban reconstruction plays an extremely important role in judging the site selection of priority reconstruction projects. The formula for calculating the potential of urban land parcel projects to be evaluated is as follows:

(5) $$\begin{array}{c} p_{i}=\sum_{j=1}^{n}a_{j}Potential_{ij}, \end{array}$$

where *P*_*i*_ is the potential value of the *i* plot to be evaluated, *a*_*j*_ is the index weight of the *j* index, and the standardized index value of the *j* index of the *i* plot.

A multi-factor comprehensive evaluation method is used to analyze and evaluate the urgency of renewal projects. The calculation formula of the urgency of the plot project to be evaluated is as follows:

(6) $$\begin{array}{c} u_{i}=\sum_{j=1}^{n}b_{j}, \end{array}$$

where *u*_*i*_ is the urgency of the *i* plot project to be evaluated, *b*_*j*_ is the index weight of the *j* index, and the standardized index value of the *j* index of the *i* plot project.

Due to limited renovation funds and other reasons, it is impossible to renovate all updated plots in a short period of time, so it is necessary to limit the total area of the plots that have priority for renovation, namely,

(7) $$\begin{array}{c} \sum_{i=1}^{n}x_{i}c_{i}\leq S, \end{array}$$

where *c*_*i*_(*i*=1,2,3,…, *n*) is the area of each plot and *S* is the priority transformation mode.

That is, *S* should meet the following conditions in quantity.

(8) $$\begin{array}{c} \sum_{i=1}^{n}x_{i}c_{i}\leq 1500. \end{array}$$

In the genetic algorithm, it is very important to determine fitness function. Selection, also known as replication, is the process of selecting excellent individuals in population to produce new population. The main body of biological evolution is population, and the calculation object of genetic calculation is also a set composed of individuals, that is, population. The operation and solution process of the genetic algorithm is very similar to the evolution process of biological natural selection. It is an iterative evolution process from generation to generation. We calculate the fitness of individuals through fitness function, and divide proportion on the roulette according to the fitness. Each individual is like a sector part of the disc. We put a pointer on the roulette for random selection. The greater the individual fitness, the greater the probability of being selected, and the smaller the fitness, the smaller the probability of being selected. Generally speaking, there are three common methods to solve optimal solution: enumeration method, heuristic method, and search method. Because the types of problems are different and the scale of problems is also different, it is unrealistic and difficult to find a general method to solve all optimization problems. However, the genetic algorithm can provide us with a practical and effective way and a relatively general and universal model and create a global heuristic optimization search algorithm.

### 3.2. Content of Protection and Inheritance of Traditional Culture in Urbanization

China has a cultural awareness of advocating nature since ancient times. Influenced by Chinese traditional culture, it believes that the Earth is an organic natural body, of which human beings are only a part. Therefore, in rural site selection and the formation of rural texture under the concept of environmental protection, people are mostly integrated into nature and live with nature according to natural conditions. The coordinated development of new urbanization also requires the integration of nature and humanities, and the combination of modern elements and traditional culture. In new urbanization, we advocate the concept of environmental protection, respect for nature, and conform to nature, which embodies the concept of harmony between man and nature. In terms of landscape, relying on the unique natural scenery in rural areas at present, let new towns integrate into nature. Using the natural environment conditions, it can be roughly summarized into three types of site selection: along the river, by the mountain, and by the lake, so that the layout of the countryside is well integrated with the natural landscape, which has been passed down to this day by the long river of time. In the protection and inheritance of excellent traditional culture in rural areas, professionals should emancipate their minds and engage in this work in a way that keeps pace with the times. The reason why culture can still be preserved in the changes of the millennium depends on the spread of the spirit and core of the environmental protection concept, and some forms of changes will not destroy its intrinsic value. In order to realize the great development and prosperity of rural cultural undertakings and the sustainable development of rural cultural industries, it is necessary to develop various technologies and equipment dedicated to rural culture and art with various environmental protection concepts, so as to provide a technical and benefit platform for rural environmental protection cultural industries.

Excellent traditional culture is the embodiment of regional soft power and the basis of national identity, national cohesion, innovation, and development. We should pay attention to its influence and constantly explore the path of inheritance and development of traditional culture. The relevance between tradition and modernity makes the renewal process more natural and coherent, so as to better solve the inheritance of local history and culture and integration with modern society. In the process of renewal and development, the main context and constituent elements of rural texture should be organically renewed on the basis of respecting the original texture and structure, so as to maintain the original rural characteristics. It is worth noting that we should pay attention to three principles in the inheritance of traditional culture under the concept of environmental protection. The protection and restoration of existing ancient relics and ancient buildings should pay attention to the authenticity, repair the old as the old, and try not to destroy the traditional cultural value contained therein. Integrity is to consider the overall environment as much as possible in the protection of historical buildings and traditional villages. Integration is the integration of nature and humanities, modernity and tradition in the protection, and inheritance of the overall traditional culture. The protection of important ancient buildings in rural areas, especially historical and cultural heritage, should be consistent with the local traditional context. For some important residential buildings and historical relics, specific environmental protection plans should be made to ensure reasonable implementation. On this basis, we should deeply explore the historical knowledge behind it, so as to create a local cultural card. Therefore, some innovative cultural protection behaviors should be supported as appropriate. For example, Kaifeng rural areas can also promote some tourism peripheral products through e-commerce platforms, and use group purchase, discount, etc. to promote the increase of tourist flow in the scenic spot. In the process of the era of the environmental protection concept, it is also necessary to pass on some ancient civilizations by “following the fashion”.

## 4. Simulation and Analysis

Generally speaking, urbanization has been developing at a high speed since the reform and opening up. According to the official data released by a province from 2016 to 2021, this paper conducted an experiment on the urbanization rate and its growth rate. The experimental results are shown in Figure 3.

As can be seen from Figure 3, the urbanization rate of a province increased from 8.9% to 28% from 2016 to 2021, with an average annual increase of about 1.25 percentage points. The total urban population increased from 6.23 million in 2016 to 48.51 million in 2021, with an average annual growth of 998000. The per capita GDP increased from 324 yuan in the early stage of reform and opening up to 5958 yuan in 2021. A series of data show that the urbanization of the province has occupied a pivotal position in the economic construction of the whole society.

In 2021, the main economic indicators of a province were analyzed experimentally, as shown in Table 1.

It can be seen from Table 1 that the economy of a province continues to maintain a steady and rapid development rate, and the GDP of the province has reached 4524.175 billion yuan, an increase of 10.8 percentage points compared with 2018. The industrial structure was further optimized. In 2021, the proportion of three industrial structures in the province was 8.8 : 53.6 : 37.3.

A genetic algorithm is used to calculate the landscape pattern index of urban construction land in a municipal area from 2018 to 2021, so as to analyze the landscape pattern characteristics of urban construction land expansion in a municipal area. Among them, LPI represents the proportion of the largest patch area of urban construction land in the total area, Contag represents the spatial aggregation degree of urban construction land, and Shei represents the balance of urban construction land distribution. The landscape pattern index of urban construction land is shown in Table 2.

As can be seen from Table 2, the number of patches of urban construction land in a municipal area gradually increased from 2018 to 2021 and decreased from 2020 to 2021, indicating that in the rapid development stage of 2018–2020, the expansion of urban construction land in a municipal area is mostly regional development, resulting in an increasing number of patches. After 2020, the development mode was gradually adjusted, the urban spatial layout was optimized, the regional development was made more centralized and balanced, and the number of fragmented patches was reduced.

Three regions for experimental analysis were selected, namely Shandong, Guangdong, and Hebei, and carried out experiments on their urbanization rate from 2016 to 2021. The experimental results are shown in Figure 4.

It can be seen from Figure 4 that the urbanization rate of three regions showed an increasing trend from 2016 to 2021, with an average annual growth rate of 1.25%. In 2018, the population urbanization rate of Shandong Province reached 53.2%, exceeding the national average. With the increase of urbanization rate, the quality of urbanization development is also improving. The factors closely related to urbanization, such as population employment, economic development, urban construction, residents' life, social development, and ecological environment, have developed harmoniously in the process of urbanization, and urbanization has entered a stage of high-quality development.

The simulation benchmark data selected in this study is the land use data of a municipal area in 2021. Taking the simulation from 2019 to 2021 as the benchmark, the initial weight is calculated to simulate the expansion of urban construction land in a municipal area from 2019 to 2021. The area statistics of various land use types in a municipal district in 2019, 2020, and 2021 are shown in Table 3.

As can be seen from Table 3, on the whole, more than 91% of the land in a municipal district is covered by cultivated land, woodland, and grassland, of which woodland occupies the largest area, and even after the rapid development in the 11th five-year plan and the 12th five-year plan, its proportion has remained stable at 35%, followed by grassland, which has remained stable at about 33.5%, making it a veritable forest city. After fifteen years of development, it gradually increased to nearly 5%. During the 12th five-year plan period, the area of urban construction land in a municipal district increased by about 25%, with an obvious growth rate and remarkable achievements in the development of new urbanization.

From 2016 to 2021, this experiment used ant colony algorithm, data mining algorithm, particle swarm optimization algorithm, and genetic algorithm to study the expansion rate of urban construction land. The experimental results are shown in Figure 5.

As can be seen from Figure 5, from the perspective of expansion rate, the growth rate from 2016 to 2021 showed the characteristics of first increasing and then decreasing. From 2016 to 2019, the expansion rate of urban construction land under the genetic algorithm reached 12% at the fastest, followed by 10% under the particle swarm algorithm, while the ant colony algorithm and data mining algorithm were only about 7% and 1%, respectively. It can be seen that the genetic algorithm in this paper is important in the expansion rate of urban construction land.

From 2016 to 2021, the accuracy of urban construction land expansion was studied by ant colony algorithm, data mining algorithm, particle swarm optimization algorithm, and genetic algorithm. The experimental results are shown in Figure 6.

As can be seen from Figure 6, among the accuracy of urban construction land expansion, during 2018, the accuracy of the ant colony algorithm for urban construction land expansion was 58%, the accuracy of the data mining algorithm was 51.8%, the accuracy of the particle swarm optimization algorithm was 56.7%, and the accuracy of the genetic algorithm in this paper was as high as 58.8%. It can be seen that the accuracy of the genetic algorithm in urban construction land expansion is the highest.

This experiment is still in 2016–2021. Ant colony algorithm, data mining algorithm, particle swarm optimization algorithm, and genetic algorithm are used to study the growth rate of urban construction land expansion. The experimental results are shown in Figure 7.

As can be seen from Figure 7, in the growth rate of urban construction land expansion, during 2019, the growth rate of urban construction land expansion of the ant colony algorithm is 35.6%, the growth rate of the data mining algorithm is 35.2%, the growth rate of the particle swarm optimization algorithm is 36.2%, and the growth rate of the genetic algorithm in this paper is 42.1%. It can be seen that the growth rate of the genetic algorithm in urban construction land expansion is the highest and shows an increasing trend.

## 5. Conclusions

To sum up, this paper studies the traditional culture of urbanization construction based on the genetic algorithm under the concept of environmental protection. Among the accuracy of urban construction land expansion, in 2018, the accuracy of the ant colony algorithm for urban construction land expansion was 58%, that of the data mining algorithm was 51.8%, that of the particle swarm optimization algorithm was 56.7%, and that of the genetic algorithm in this paper was as high as 58.8%. It can be seen that the genetic algorithm in this paper has the highest accuracy in the expansion of urban construction land. On the practical level, urbanization construction through the genetic algorithm should pay special attention to the concept of environmental protection, the inheritance and embodiment of cultural traditions, and advocate the establishment of a constructive development concept characterized by showing uniqueness with an open concept, so as to build a colorful world where constructive development and culture coexist harmoniously. In China, villages are earlier than cities, and their emergence and development have certain rules to follow, which endows them with profound historical accumulation. If we want to protect history and culture under the concept of environmental protection, we must clearly show it and let it continue to develop healthily, so as to achieve the purpose of protection. In the process of development, it should be noted that urban and rural areas are different spatial areas, which must have different characteristics and respective advantages. In order to realize the great development and prosperity of rural cultural undertakings and the sustainable development of rural cultural industries, it is necessary to develop various technologies and equipment dedicated to rural culture and art with various environmental protection concepts, so as to provide a technical and benefit platform for rural environmental protection cultural industries.

## Figures and Tables

**Figure 1:** Flow chart of the genetic algorithm.

**Figure 2:** Model diagram of traditional cultural structure in urbanization construction.

**Figure 3:** Changes in the urbanization rate and urbanization rate growth of a province from 2016 to 2021.

**Figure 4:** Urbanization rate trend in different regions from 2016 to 2021.

**Figure 5:** Trend of urban construction land expansion rate with different algorithms.

**Figure 6:** Accuracy of urban construction land expansion with different algorithms.

**Figure 7:** Growth rate of urban construction land expansion with different algorithms.

**Table 1:** List of main economic indicators of a province in 2021.

Total index	Numerical value	GPer capita index growth rate	Per capita index	Numerical value	Growth rate
GDP	45241.75	10.8	Per capita GDP	47334	10.1
Added value of secondary industry	24016.12	11.6	Per capita local general budget revenue	3591.21	24.62
Added value of secondary industry	17370.88	11.2	Energy consumption per 10000 yuan GDP	0.85	−3.76
Total imports and exports	2359.91	24.8	Dependence on foreign trade	33.5	0.8

**Table 2:** Landscape pattern index of urban construction land in a municipal district from 2016 to 2021.

Particular year	NP	LPI	Contag	Shei
2018	496	96.978	88.512	0.194
2019	527	96.835	88.104	0.203
2020	561	96.165	86.412	0.231
2021	473	96.016	85.887	0.241

**Table 3:** Area statistics of land use types from 2019 to 2021.

Category	2019		2020		2021	
	Area	Proportion	Area	Proportion	Area	Proportion
Woodland	924.436	36.082	1308.427	36.094	1308.082	36.084
Urban construction land	109.133	3.012	114.262	3.151	137.308	3.787
Unused land	1.273	0.036	1.273	0.034	1.273	0.034

## Data Availability

The data used to support the findings of this study are available from the corresponding author upon request.
